The article "Innate Immune Activation by Inhaled Lipopolysaccharide, Independent of Oxidative Stress, Exacerbates Silica-Induced Pulmonary Fibrosis in Mice" was retracted in 2016. Reasons: errors in the data; errors in the methods; unreliable data; concerns about the data.

# Innate Immune Activation by Inhaled Lipopolysaccharide, Independent of Oxidative Stress, Exacerbates Silica-Induced Pulmonary Fibrosis in Mice

**DOI:** 10.1371/journal.pone.0040789

**Published:** 2012-07-16

**Authors:** David M. Brass, Jennifer C. Spencer, Zhuowei Li, Erin Potts-Kant, Sarah M. Reilly, Mary K. Dunkel, Joseph D. Latoche, Richard L. Auten, John W. Hollingsworth, Cheryl L. Fattman

**Affiliations:** 1 Neonatology Division, Department of Pediatrics, Neonatal Perinatal Research Institute, Duke University Medical Center, Durham, North Carolina, United States of America; 2 Pulmonary Allergy and Critical Care Division, Department of Medicine, Duke University Medical Center, Durham, North Carolina, United States of America; 3 Department of Environmental and Occupational Health, University of Pittsburgh Graduate School of Public Health, Pittsburgh, Pennsylvania, United States of America; 4 Department of Immunology, Duke University Medical Center, Durham, North Carolina, United States of America; French National Centre for Scientific Research, France

## Abstract

Acute exacerbations of pulmonary fibrosis are characterized by rapid decrements in lung function. Environmental factors that may contribute to acute exacerbations remain poorly understood. We have previously demonstrated that exposure to inhaled lipopolysaccharide (LPS) induces expression of genes associated with fibrosis. To address whether exposure to LPS could exacerbate fibrosis, we exposed male C57BL/6 mice to crystalline silica, or vehicle, followed 28 days later by LPS or saline inhalation. We observed that mice receiving both silica and LPS had significantly more total inflammatory cells, more whole lung lavage MCP-1, MIP-2, KC and IL-1β, more evidence of oxidative stress and more total lung hydroxyproline than mice receiving either LPS alone, or silica alone. Blocking oxidative stress with N-acetylcysteine attenuated whole lung inflammation but had no effect on total lung hydroxyproline. These observations suggest that exposure to innate immune stimuli, such as LPS in the environment, may exacerbate stable pulmonary fibrosis via mechanisms that are independent of inflammation and oxidative stress.

## Introduction

The factors that contribute to the pathogenesis and progression of fibrotic lung disease remain poorly understood. Fibrotic lung disease may be caused by inhalation of organic or inorganic substances, by medications or infection; may be associated with clinical conditions such as connective tissue disease; or may be idiopathic in nature. Rates of incidence and prevalence of fibrotic lung diseases are difficult to estimate, although a recent study shows that incidence can range between 19.4 and 34.3 per 100,000 [1]. In particular, exposure to crystalline silica in occupational settings has historically been estimated to be in the millions annually in the US alone [2] and thus continues to be a significant occupational risk factor. We use crystalline silica instillation in mice as a clinically relevant model of human disease because silica instillation leads to lung injury that is consistent and uniformly similar with pulmonary lesions observed in patients with occupational silicosis.

Broadly, fibrotic lung diseases may be characterized as slowly progressing, rapidly progressing or punctuated by episodes of disease acceleration known as acute exacerbations [3]. It is increasingly recognized that a significant portion of the population with interstitial lung diseases that develop lung fibrosis suffer from episodes of accelerated disease progression for unknown reasons [4], [5], [6]. Acute exacerbations of pulmonary fibrosis occur in approximately 14% of patients with idiopathic pulmonary fibrosis each year [7]. The differences between slowly and rapidly progressing fibrotic lung disease are becoming somewhat more clear [8] although the causes for these differences remain obscure. Similarly, the causes of acute exacerbations of lung fibrosis remain to be determined. First described in 1993 [9], the definition of an acute exacerbation has come to include 1) increased dyspnea within 1 month; 2) hypoxemia; 3) new pulmonary infiltrates that are visible by radiography; and 4) absence of infection or evidence of a cardiac event [10]. The idiopathic and apparently stochastic nature of acute exacerbations renders them very difficult to study. Nevertheless, some attempts have been made to identify mechanisms that could contribute to such exacerbation events. For example, viral infections have frequently been observed in cases of lung fibrosis [11], and viral accelerations of lung fibrosis have been successfully modeled in mice and are characterized by Th1 cytokine and fibrogenic growth factor expression that is consistent with activation of innate immunity [12], [13]. Viral particles are recognized by Pathogen Associated Molecular Pattern (PAMP) receptors in the Toll-Like Receptor (TLR) family and are able to activate an innate immune response in the lung. We have previously shown that innate immune stimulation of the lung with the canonical activator of innate immunity, lipopolysaccharide (LPS), can increase expression of genes commonly associated with lung fibrosis and can induce fibroproliferative airway remodeling [14]. Therefore, our overall hypothesis is that environmental exposures that activate innate immunity contribute to acceleration of or exacerbation of stable pulmonary fibrosis. To address this hypothesis, we first exposed mice to crystalline silica in the lung and 28 days later, exposed these mice to LPS by aerosol inhalation. Our observations suggest that exposure to LPS, or other common environmental exposures that activate innate immunity, could contribute to acceleration of, or acute exacerbations of fibrotic lung disease in patients with pulmonary fibrosis.

## Materials and Methods

### Animals and Exposures

Eight week old male C57BL/6 male mice (Jackson Laboratory, Bar Harbor, ME) were given a single oropharyngeal aspiration of 0.2 g/kg crystalline silica (Min-U-Sil 5 [15], [16]; a generous gift from Dr. Andy Ghio, US Environmental Protection Agency) in 60 µl of sterile 0.9% saline or an equivalent volume of 0.9% saline alone at day 0. On day 28, groups of mice (n = 6/group) were then either exposed to an aerosol of LPS as previously described [17] at a target concentration of 0.5 µg/m^3^ or to an aerosol of sterile 0.9% saline for 2.5 hours per day for five consecutive days under barrier conditions. Groups of mice were then sacrificed immediately after the end of the last LPS exposure or were allowed to recover for 21 days before sacrifice. Treatment groups are referred to by exposures in the order administered. ***Saline-Saline*** first received the vehicle control for silica via oropharyngeal aspiration followed 28 days later by the aerosolized saline control for LPS; ***Saline-LPS*** first received the vehicle control for silica via oropharyngeal aspiration followed 28 days later by aerosolized LPS; ***Silica-Saline*** first received 0.2 g/kg silica via oropharyngeal aspiration followed 28 days later by the aerosolized saline control for LPS, and; ***Silica-LPS*** first received 0.2 g/kg silica via oropharyngeal aspiration followed 28 days later by aerosolized LPS. Mice treated with N-acetylcysteine (NAC) were provided with drinking water supplemented with 2 mg/ml NAC as described previously [18] for the period beginning three days prior to the start of LPS inhalation and lasting until phenotyping (n = 8/group). All animal procedures were approved by the Duke University Institutional Animal Care and Use Committee.

### Hydroxyproline Analysis

Whole lungs were lyophilized and then acid hydrolyzed in sealed, oxygen-purged glass ampules containing 2 ml of 6 N HCl at 110°C for 24 h. Samples were resuspended in 1.5 ml of phosphate buffered saline and incubate at 60°C for 1 h. Samples were centrifuged at 13,000 rpm for 10 min. and the hydroxyproline analysis was performed on the resulting supernatant using chloramine-T spectrophotometric absorbance as previously described [19].

### Lung Histology

Lung sections were stained with Masson’s trichrome to visualize collagen. Images were captured at either 5× or 20× magnification, and the color balance for each image was adjusted equally using Adobe Photoshop.

### Analysis of Bronchoalveolar Lavage Fluid (BALF)

Mice were euthanized by CO_2_ inhalation, and lungs were lavaged three times to capacity with 0.9% saline through PE-90 tubing at a pressure of 20 cmH_2_O. The collected lavage fluid was processed and stored for further analysis as previously described [20]. Total MCP-1, MIP-2 and KC concentrations in the BALF were determined using Duo-Set ELISA kits (R&D Systems; Minneapolis MN) according to the manufacturer’s instructions. Protein carbonyl content of the BALF was determined using the Cell BioLabs, Inc (San Diego, CA) OxiSelect^TM^ protein carbonyl ELISA kit according to the manufacturer’s instructions.

### Statistical Analyses

All data are expressed as means ± SE. Differences between groups and between variables were analyzed by ANOVA. Probability values of P<0.05 (two-tailed) were considered statistically significant.

## Results

### Innate Immune Stimulation Significantly Increases Total Lung Hydroxyproline Content in Mice Previously Exposed to Crystalline Silica

To address whether innate immune stimulation would contribute to pre-existing lung fibrosis, we first exposed 8 week old C57BL/6 mice to either crystalline silica or vehicle alone via oropharyngeal aspiration. This was followed 28 days later by exposure of these groups of mice to either aerosolized LPS or sterile saline. We observed that immediately and 21 days after the aerosol exposure (Figure 1) there was no difference in total lung hydroxyproline between Saline-Saline (closed square) and Saline-LPS groups (open square), indicating that LPS exposure by itself did not increase total lung hydroxyproline in these mice. Both immediately and 21 days after the aerosol exposure (Figure 1) we observed that exposure to crystalline silica by itself (Silica-Saline group, closed triangle) significantly increased total lung hydroxyproline content when compared with the Saline-Saline group. Importantly, we observed that mice exposed to both silica and inhaled LPS (Silica-LPS, open triangle) had significantly more total lung hydroxyproline than control mice exposed to saline alone (Saline-LPS), or mice exposed to silica alone (Silica-Saline). These observations taken together demonstrate that activation of the innate immune system in the lung increases total lung hydroxyproline in mice with pre-existing lung fibrosis.

**Figure 1:** Hydroxyproline content in whole lung tissue. Total hydroxyproline per lung immediately after and 21 days after the end of inhalation challenge. Data are presented as Mean + SEM and are representative of two such experiments. n = 6/group. * p<0.05 LPS vs. Saline (significant difference due to inhalation challenge); # p<0.05 Silica vs. Saline (significant difference due to silica instillation or combined Silica and LPS).

The significant increases in hydroxyproline associated with LPS inhalation challenge consequent to silica instillation may be appreciated histologically as shown in Figure 2 (immediately after) and Figure 3 (21 days after). We observed that immediately after either saline or LPS inhalation challenges (Saline-Saline and Saline-LPS groups; Figures 2A & 2C) there were no significant histological differences between groups. However, in the Silica-Saline group, immediately after the end of saline inhalation challenge we observed prominent areas of inflammation and loosely organized fibrotic tissue (Figure 2B). Importantly, in the Silica-LPS group immediately after the end of the LPS inhalation challenge, we observed a greater overall degree of fibrosis and the presence of enlarged macrophages with diffusely transparent cytoplasm (Inset in Figure 2D) consistent with pulmonary alveolar proteinosis [21]. While these macrophages were observed in the Silica-Saline group, their presence was more prominent in the Silica-LPS group.

**Figure 2:** Histology immediately after the end of inhalation challenge. (A) Saline-Saline; (B) Silica-Saline; (C) Saline-LPS; and (D) Silica-LPS exposed mice immediately after the end of either saline or LPS inhalation challenge. n = 6/group. Images were taken in anatomically comparable regions of the lung at 5× (main images) or 20× (Inset in panel D) magnification. Bar = 100 microns.

**Figure 3:** Histology 21 days after the end of inhalation challenge. (A) Saline-Saline; (B) Silica-Saline; (C) Saline-LPS; and (D) Silica-LPS exposed mice immediately after the end of either saline or LPS inhalation challenge. n = 6/group. Images were taken in anatomically comparable regions of the lung at 5× (main images) or 20× (Inset in panel D) magnification. Bar = 100 microns.

Similarly, at 21 days after the end of inhalation challenge there were no apparent differences between the Saline-Saline and Saline-LPS groups (Figures 3A & 3C). As with the mice sacrificed immediately after the end of inhalation challenge, we observed prominent areas of inflammation and consolidated fibrotic tissue in mice in the Silica-Saline group (Figure 3B). In the histological sections from the Silica-LPS group mice sacrificed 21 days after the end of inhalation challenge, we observed notable areas of condensed fibrotic tissue with prominent collagen staining (Figure 3D). We also observed the persistent presence of enlarged macrophages with diffusely transparent cytoplasm (Inset in Figure 3D) in this group of mice.

### Innate Immune Stimulation in Mice Previously Exposed to Crystalline Silica Causes a Significantly Increased Inflammatory Response

As we and others have previously observed [17], [22], exposure to inhaled LPS alone (Saline-LPS, open square) causes an immediate significant increase in total lung inflammatory cells when compared to mice exposed to aerosolized saline (Saline-Saline, closed square) (Figure 4A). Consistent with previous observations, we show here that the majority of the inflammatory cells recruited to the lung in response to inhaled LPS are polymorphonuclear leukocytes (PMNs) (Figure 4C), although there are also significant increases in total lung macrophages (Figure 4B) and lymphocytes (Figure 4D). We also observed that, consistent with previous reports [23], silica exposure alone (Silica-Saline, closed triangle) significantly increased total lung inflammatory cells (Figure 4A), of which equal numbers are PMNs (Figure 4C) and macrophages (Figure 4B) while total lung lymphocytes are also increased (Figure 4D). Notably, prior exposure to silica significantly increases the immediate inflammatory response to inhaled LPS (Silica-LPS, open triangle; Figure 4A) with the majority of the additional cells recruited also being PMNs (Figure 4C; also compare Figure 4B Silica-Saline and Silica-LPS showing no increase in total lung macrophages resulting from the combined exposure). At 21 days after LPS exposure the immediate cellular inflammatory response to inhaled LPS alone (Saline-LPS) resolves completely (Figure 4A showing total cells and 4C showing total PMNs). Consistent with previous reports there is still a significant inflammatory response to silica exposure alone (Silica-Saline) that is comprised of macrophages, PMNs and lymphocytes (Figure 4A–D). Importantly, in mice exposed to both silica and LPS (Silica-LPS) the effects of the combined exposure cause a significant and persistent increase in total cellular inflammation in the lung (Figure 4A). The total number of macrophages in this group is also significantly increased when compared to total number of macrophages recruited by silica exposure alone (Silica-Saline).

Consistent with the cellular response we also observed that the pro-inflammatory cytokines MCP-1, MIP-2 and KC, that are known to recruit macrophages (MCP-1) and neutrophils (MIP-2 and KC) to sites of ongoing inflammation, are similarly increased in whole lung lavage fluid immediately after the end of the aerosol exposure (Figure 5). Interestingly, IL-1β which we have previously shown to be increased by LPS inhalation alone [17] is not significantly increased by combined exposure to silica and LPS at this time point (Figure 5D). Notably, at 21 days after the aerosol exposure total MCP-1 in whole lung lavage fluid remains significantly increased in the Silica-LPS group when compared to the Silica-Saline group at this time point (Figure 5A). There is no difference between these groups in total MIP-2 or IL-1β at this time point. These observations taken together show that innate immune stimulation causes a significant and persistent increase in whole lung inflammation in mice with pre-existing silica-induced lung fibrosis.

**Figure 4:** Whole lung lavage immediately after and 21 days after the end of inhalation challenge. (A) Total cells×10^5^; (B) total macrophages×10^5^; (C) total neutrophils×10^5^; and total lymphocytes×10^5^. Data are presented as Mean + SEM and are representative of two such experiments. n = 6/group. * p<0.05 LPS vs. Saline (significant difference due to inhalation challenge); # p<0.05 Silica vs. Saline (significant difference due to silica instillation or combined Silica and LPS).

**Figure 5:** Whole lung cytokines immediately after and 21 days after the end of inhalation challenge. Total (A) MCP-1; (B) MIP-2; (C) KC; and (D) IL-1β in whole lung lavage. Data are presented as Mean + SEM and are representative of two such experiments. n = 6/group. * p<0.05 LPS vs. Saline (significant difference due to inhalation challenge); # p<0.05 Silica vs. Saline (significant difference due to silica instillation or combined Silica and LPS).

To investigate the role of oxidative damage resulting from exposure to silica and to LPS we measured the concentration of protein carbonyls in whole lung lavage fluid [24], [25]. We observed that by themselves neither prior silica exposure (Silica-Saline) nor LPS exposure (Saline-LPS) caused an increase in protein carbonyl concentration in whole lung lavage fluid. However, combined exposure to both silica and LPS (Silica-LPS) resulted in a significant increase in protein carbonyl concentration in whole lung lavage fluid immediately after LPS exposure (Figure 6). By 21 days after the LPS exposure there was no difference in the concentration of protein carbonyls in whole lung lavage fluid between any of the groups (Figure 6). These observations taken together suggest that oxidative stress resulting from exposure to inhaled LPS in the context of pre-existing silica-induced lung fibrosis could be contributing to the increased collagen deposition seen both immediately after and 21 days after LPS exposure in Silica-LPS mice.

**Figure 6:** Protein carbonyls in whole lung lavage protein. Concentration of protein carbonyls in whole lung lavage protein immediately after and 21 days after the end of inhalation challenge is shown. Data are presented as Mean + SEM and are representative of two such experiments. n = 6/group. * p<0.05 LPS vs. Saline (significant difference due to inhalation challenge); # p<0.05 Silica vs. Saline (significant difference due to silica instillation or combined Silica and LPS).

### Blocking Oxidative Stress with N-acetylcysteine during LPS Inhalation Attenuates Inflammation but not Fibrosis

To investigate the role of oxidative stress resulting from exposure to silica and to LPS we exposed groups of mice to silica and then to either inhaled saline or LPS as before. Groups of mice were given either normal drinking water or drinking water supplemented with 2 mg/ml of N-acetylcysteine (NAC), which has previously been shown to block oxidative stress and to protect from oxidative stress-induced airspace enlargement [18], prior to and during LPS inhalation challenge. We observed that blocking oxidative stress with NAC failed to protect from the enhanced fibrosis caused by LPS inhalation challenge in silica-exposed mice (Figure 7). However, NAC treatment prior to and during LPS inhalation significantly reduced the total inflammatory response (Figure 8A) by attenuating the recruitment of PMNs (Figure 8C) while the total numbers of macrophages and lymphocytes was unchanged. NAC treatment significantly reduced the macrophage chemoattractant chemokine MCP-1 (Figure 9A), but not the neutrophil-specific chemoattractant chemokines MIP-2 (Figure 9B) or KC (Figure 9C). Interestingly, NAC treatment significantly reduced the amount of IL-1β (Figure 9D) present in whole lung lavage fluid.

**Figure 7:** Hydroxyproline content in whole lung tissue in mice treated with drinking water alone or drinking water supplemented with 2 mg/ml NAC during LPS exposure. Data are presented as Mean + SEM. n = 8/group. * p<0.05 LPS vs. Saline (significant difference due to inhalation challenge).

**Figure 8:** Whole lung lavage immediately after the end of inhalation challenge in mice treated with drinking water alone or drinking water supplemented with 2 mg/ml NAC during LPS exposure. (A) Total cells×10^5^; (B) total macrophages×10^5^; (C) total neutrophils×10^5^; and (D) total lymphocytes×10^5^. Data are presented as Mean + SEM. n = 8/group. * p<0.05 LPS vs. Saline (significant difference due to inhalation challenge); ^∧^ p<0.05 vs. regular drinking water (significant difference due to NAC treatment alone); # p<0.05 Silica vs. Saline (significant difference due to silica instillation or combined Silica and LPS).

**Figure 9:** Whole lung cytokines immediately after the end of inhalation challenge in mice treated with drinking water alone or drinking water supplemented with 2 mg/ml NAC during LPS exposure. Total (A) MCP-1; (B) MIP-2; (C) KC; and (D) IL-1β in whole lung lavage. Data are presented as Mean + SEM. n = 8/group. * p<0.05 LPS vs. Saline (significant difference due to inhalation challenge); # p<0.05 Silica vs. Saline (significant difference due to silica instillation or combined Silica and LPS).

## Discussion

We have shown that innate immune stimulation with LPS in the context of pre-existing silica-induced lung fibrosis either accelerates or exacerbates the existing disease. This is accompanied by significant increases in cellular inflammation at both time points examined and concomitant increases in pro-inflammatory cytokine production. Furthermore, this is accompanied by evidence that only combined exposure to both silica and LPS leads to an increase in evidence of oxidative damage to proteins in whole lung lavage fluid. However, blocking oxidative stress during the LPS exposures failed to attenuate the observed LPS-induced increases in hydroxyproline. These observations taken together provide evidence that exposure of the lung to LPS, which is ubiquitous in the environment, could lead to exacerbations or acceleration of disease progression in patients with stable pulmonary fibrosis. They further suggest that anti-oxidant therapy in vulnerable patients could reduce inflammation associated with such exacerbations but that this treatment would likely have limited effect on loss of normal lung architecture.

The pathogenesis of pulmonary fibrosis remains poorly understood [26]. This is due in large part to the obvious challenge presented by the study of human end stage disease that may not reveal the mechanistic early events that lead to later development of fibrosis. An additional challenge is the lack of similarity of common disease models with human lung fibrosis. Silica is a biologically relevant fibrogenic environmental dust and the resulting pathology in mice has many features in common with human silicosis. The silica model gives us the opportunity to study both early and late stage events in development of experimental lung fibrosis and to use this model to understand how common environmental exposures may accelerate or exacerbate existing disease in human patients. Our data show that activation of innate immunity by LPS in mice previously exposed to crystalline silica enhances many previously observed features of human silicosis including inflammation, evidence of oxidative stress-induced lung damage, collagen deposition and the presence of enlarged foamy macrophages that are consistent with pulmonary alveolar proteinosis [21], [27]. While we observed enlarged foamy macrophages most prominently in the Silica-LPS groups both immediately after and 21 days after the end of the aerosol challenge it is unclear what the role of these cells may be in the disease process. Our observations taken together support our previously published observations [14] and other studies [28], [29] showing that LPS inhalation by itself induces many genes that are also induced in experimental fibrosis. Importantly, the current observations showing that blocking oxidative stress with NAC blocks inflammation but not fibrosis exacerbation supports the notion that inflammation and fibrosis are at least partially independent processes [30], [31], [32], [33], [34].

Interestingly, the role of inflammation in development and progression of lung fibrosis remains controversial. For example, a recent study has demonstrated that nucleotide-binding domain and leucine-rich repeat containing (NLR) protein family member 3 (Nalp3)-dependent pro-inflammatory mediators are critical to development of lung fibrosis in the silica model [35] and these multi-protein complexes contribute significantly to development of inflammation. Interestingly, recent studies have demonstrated that innate immune activation may play a central role in the response to crystalline silica [36] and that macrophages in particular may drive the complete response to silica in the lung through the inflammasome [35], [36], [37].

In general, inflammasomes sense both exogenous and endogenous danger signals through intracellular NOD-like receptors (NLRs) [38] that activate caspase-1 which in turn promotes cleavage and activation of the pro-inflammatory cytokine IL-1β [38], [39]. Previous studies have shown the importance of IL-1β in the response to crystalline silica exposure. Silica-treated macrophages secrete IL-1β, and IL-1β-deficient mice have an altered inflammatory response to silica [40], [41]. In addition, a polymorphism in the gene encoding the endogenous receptor antagonist for the IL-1 receptor (IL-1Ra) has been associated with increased susceptibility to silicosis in a human population [42]. Silica exposure activates the inflammasome [43] and Nlrp3 deficient mice are protected from the effects of silica in the lung [35] suggesting that the inflammasome is critical to a complete *in vivo* response to silica. LPS has also been shown to activate the inflammasome, and mice deficient in Caspase-1, a key component of the inflammasome, have a primary defect in the ability to produce and secrete IL-1β in response to LPS [44]. We therefore hypothesized that LPS exposure would significantly enhance IL-1β protein concentrations in whole lung lavage fluid over the concentrations induced by silica exposure and that this could be causally linked to the observed increases in fibrosis. However, our observations demonstrate clearly that LPS inhalation challenge failed to enhance IL-1β concentrations in whole lung lavage over silica alone. Blocking oxidative stress with NAC fails to protect from the enhanced fibrosis seen in mice exposed to both silica and inhaled LPS. NAC treatment significantly attenuated inflammation and the concentration of IL-1β in whole lung lavage fluid in mice exposed to both silica and LPS while having no effect on hydroxyproline content of the lung. These observations are consistent with previous reports showing that inhibitors of reactive oxygen species (ROS) inhibit IL-1β secretion [35], [45]. LPS inhalation exposure, by itself, can increase ECM gene expression [14] and therefore, exacerbation or acceleration of fibrosis observed in Silica-LPS mice may be a result of direct innate immune stimulation of ECM gene expression rather than being a by-product of enhanced inflammation.

In summary, we have demonstrated that inhalation of the TLR4 ligand LPS, exacerbates or accelerates silica-induced fibrotic lung disease. This was associated with increases in total lung inflammation and in cytokines and chemokines that are chemoattractants for macrophages and neutrophils. Additionally we have shown that only mice exposed to both silica and LPS have significant increases in evidence of oxidative damage in the lung but that blocking oxidative stress with NAC fails to attenuate the enhanced hydroxyproline deposition observed in mice exposed to both silica and LPS. These data suggest that inhalation of environmental LPS and possibly other TLR ligands may contribute to exacerbation or acceleration of pre-existing disease in patients with pulmonary fibrosis in a manner that is independent of inflammasome activation or inflammation.
